This article has been retracted.

# Semantic Construal Mechanism of the Linguistic Environment Parameter Theory in Business English Translation

**DOI:** 10.1155/2022/8953181

**Published:** 2022-07-20

**Authors:** Xin Li

**Affiliations:** Yinchuan University of Energy, Yinchuan 750001, China

## Abstract

The theory of linguistic environment parameters has an important influence on English translation. Based on this parameter, it can provide guidance for the semantic generation of English translation. In the actual translation process, people's native language thinking amount accounts for 56.2% and English thinking amount accounts for 43.8%. Translation is mostly used in texts, accounting for 40.6%, and thinking based on the context parameter theory accounts for only 3.2%. To a certain extent, it can be seen that people's thinking about business English translation will be affected by different amounts of thinking. By mapping context parameters to corresponding factors, this paper analyzes the interpretation mechanism of translation semantics, to a certain extent, more intuitively expounds the semantic generation of business English translation, puts forward higher requirements for people's translation ability, and further obtains new knowledge, so as to provide practical guidance for English translation.

## 1. Introduction

Business English covers a wide range of content, including international trade, marketing, and other fields. Therefore, the translation objects of business English are diversified, and different professional fields have different requirements for the language system of translation. If you want to do a good job in English translation, you should not only have the comprehensive ability of reading and understanding, but also necessarily explore the regular characteristics of the translation of various words, so as to provide valuable references for translation [1]. Common words in the context of business English will be given new meanings. This requires translators to fully grasp the use of vocabulary and translation methods, give full play to the function of the semantic construal mechanism, and further improve the translation mechanism. Genre is an example of communicative activities that achieve specific goals by using conventional language and discourse knowledge. Each genre constructs a narrow experience or real-world experience in a specific way, which is recognized and understood by members of its professional field. Stylistic function refers to the unique meaning given by the author to the language order of a work (text) and to the effectiveness of this meaning to the reader; the effect of stylistic function is closely related to the language used by the author and the language in the specific context. Grammatical metaphor is a process in which the author reselects the language system (meaning system and lexical grammar system) in the context of the situation. It is an important means and resource for the author to endow his works (texts) with a unique meaning. In the process of discourse construction, the characteristic of grammatical metaphor lies in the condensation of meaning, the construction of “imaginary or imaginary things,” and the unique function of “name is not name, but called it” [2]. At the context level, business English contract and letter communication are two common sub categories in the international business language category, and they are also two key links in the process of international business communication. The former provides a guarantee for the orderly development of international business communication, and the latter runs through the whole process of international business communication. At the textual level, compared with general English, business English contracts and letters are highly grammatical metaphorical professional texts, but there are also some stylistic differences between them. These stylistic differences may be related to the use of grammatical metaphors. The topic of this study not only helps to enrich the research content of the theoretical system of grammatical metaphors, but also broadens the vision of business English research and boosts the development of business English linguistics [3].

## 2. Genre and Style

Before introducing business English, business English contracts, and business English letters, we need to trace their upper-level categories, categories, and styles, so as to have a macro grasp of them, involving their concepts, characteristics, and relationships.

### 2.1. Characteristics of Category Definition

The concept of genre comes from development and is expressed as a specific artistic style according to the dictionary. After the localization of English, it has the connotation of variety and style. There are some differences in the definition of genre. The classification standard focuses more on the division of the language field, that is, the division of situational context, such as legal style, business style, and scientific and technological style. In genre culture, the cultural context is determined by symbols. The shallow potential of symbols in language constitutes the shallow potential of genre meaning, as shown in Figure 1.

### 2.2. Relationship between Genre and Style

In terms of conceptual categories, genre and style belong to two different conceptual categories. The core content of the conceptual structure of genre is the types of social and cultural activities with certain communicative purposes, which are embodied in different types of discourse. The nature of genre is determined by the potential of the meaning structure of genre. Three situational contexts, configuration elements, field, and tenor and mode, jointly restrict the choice of genre. In terms of the level of abstraction and semantic implication, the relationship between genre and style can be summarized as whole and part, abstract and concrete, and unified and special [4, 5]. The former is an abstract and generalized collective concept of the category of social and cultural activities that express unified communication goals. The latter is a series of specific linguistic features that express particularity. The former includes the latter, as shown in Figure 2.

### 2.3. Research on Business English

From the English language teaching tree (Figure 3), it can be seen that business English is regarded as a subordinate branch of English, which is juxtaposed with scientific English. The definition of business English needs to involve language knowledge and business communication skills.

According to the context view and language level view of systemic functional linguistics, business discourse should be at a level from international business discourse to international business culture: ideology (international business culture) ⟶ international business discourse ⟶ international business register ⟶ international business discourse (⟶ refers to the realization relationship; realization refers to the relationship “hierarchy of abstraction” between various abstract levels, for example, social context is realized by the language system and ideology is realized by the language category at the level of social context), as shown in Figure 4.

According to the language hierarchy, the interpretation of grammar needs to be understood according to Figure 5. Under the tension of language levels, the logical meaning originally embodied by logical connectives, the attribute feature meaning embodied by adjectives, and the process meaning embodied by verbs are all embodied by nouns, which are reinterpreted as the participant meaning.

The meaning of language metaphors needs to be transferred according to the expression of specific things. The semantic transformation to specific things is similar to the traditional lexical metaphor [6, 7].

## 3. Hypothesis of the Binary Structure Theory

### 3.1. Theoretical Basis

The cognitive learning theory attaches importance to learners' internal psychological processes. Whether various stimuli in the environment are paid attention to or processed depends on people's internal psychological structure. It is a choice made by people according to their own internal psychological structure. The individual endows experience with meaning through interaction with the environment, and organizes and reorganizes the experience, so as to modify or construct their own cognitive structure. Therefore, the study of the learning process should pay attention to the internal mechanism of learners' psychology. After being exposed to specific language knowledge, learners acquire language bit by bit through the language acquisition mechanism of the brain and the universal grammar it contains [8]. Learners slowly accumulate specific language knowledge and develop their own knowledge structure and cognitive structure, as shown in Figure 6.

### 3.2. Operation Mechanism of the Dual Structure Theory

The theory of “dual structure” holds that different languages have different characteristics and different symbol systems, so the language knowledge of people learning different languages is different, and the knowledge established is different. In the process of integrating new knowledge with old knowledge, a new structure of language cognition is formed, and in the process of cognition, a new structure and cognitive structure are formed, as shown in Figure 7.

When learners learn another language—English, they will inevitably gradually establish the English knowledge structure and English cognitive structure corresponding to English in the learning process. At this time, when learners learn new English language knowledge, the process is different from their mother-tongue acquisition, because their mother-tongue knowledge structure and cognitive structure are completely different from English in the minds of learners. At this time, a “dual structure” is formed in the minds of learners. In the process of knowledge assimilation, the “dual structure” has a dynamic relationship with each other, as shown in Figure 8.

As can be seen from the abovementioned figure, the relationship between the knowledge structure and cognitive structure of mother tongue and English has been developing in the process of assimilation, forming a new knowledge structure and cognitive structure of the mother tongue and English, that is, the process of our English learning. When it comes to language, it has always been closely related to our thinking. The essence of the knowledge structure of mother tongue and English is two languages, and the core of the cognitive structure of the two languages is our mother tongue and English thinking. Therefore, the essence of “dual structure” is the relationship between English and Chinese bilingual language and thinking [9–11].

## 4. Empirical Research

### 4.1. Research Design

From the abovementioned analysis, we can see that in the process of English reading comprehension, we not only have English thinking, but also have mother-tongue thinking. In view of this phenomenon, it is necessary to study the dependence of learners on language thinking and whether their reading ability is different under the influence of mother-tongue thinking. Fifteen non-English major freshmen from Xihua University participated in the study. All of them were from classes 3 and 4 of the School of Applied Technology, Xihua University, with an average age of 20 years. Their English study period is about 9 years, and their English scores are 118 on average. Recommended by their teachers, these students are extroverted and easy to cooperate. They are middle and upper-level English learners among similar students.

### 4.2. Research Methods and Tools

Research methods and tools include the following: thinking aloud, retrospective interviews, two CET texts, and MP3 recorders. The topics of the text are “American primary education” and “grandparent program organization,” both of which are illustrative texts (Table 1). Data were input into SPSS 12.0 for statistics.

### 4.3. Data Analysis

Data analysis materials include a voice thinking report and interview record report. The researcher makes qualitative and quantitative analyses of mother-tongue thinking in the voice thinking report. First, count the number of Chinese and English words (including repeated words) in each record and calculate the average total number of words of 15 people (first, calculate the total number of Chinese and English words when each person reads CET-4 and CET-6, and then, add the total number of words of 15 people to calculate the average number); then, calculate the number of Chinese words and English words per capita of 15 people when reading CET-4 and CET-6, respectively (for example, the number of Chinese words per capita of 15 people when reading CET-4 is added and divided by 15 to obtain the number of Chinese words per capita in CET-4). The number of Chinese words per capita can be obtained from the number of Chinese words per capita when reading CET-4 plus the number of Chinese words per capita when reading CET-6. The algorithm for the number of English words per capita is the same. The determination of Chinese words is based on the method of Wang Wenyu and Wen Qiufang (2002), that is, the modern Chinese dictionary shall prevail. The following method is the statistical method for the amount of thinking: the proportion of the average number of Chinese/English words in the average total number of words (the total number of Chinese and English words); the distribution of Chinese in each thinking activity (the average number of Chinese words in a thinking activity/the average total number of Chinese words); the proportion of the average number of Chinese/English words in the total amount of thinking in each thinking activity (mother tongue and autonomous English thinking). The following statistics are the average number of 15 people [12–14].

The quantitative analysis of 30 reading records shows that the amount of thinking in mother tongue accounts for 56.2% of the total amount of thinking; the amount of thinking in English is 43.8%, but most English is used for reading texts (40.6%), and only a small part (3.2%) is used for autonomous thinking (Table 2).

After observing the distribution of mother-tongue thinking in various reading activities (Table 3), 85.2% of mother-tongue thinking is used to construct text meaning, 7.2% and 7.6% are used to distinguish language forms and manage reading behavior, respectively. It can be seen from the table that the students are more dependent on their mother tongue, leading to their thinking activities taking the first place. It can be said that in the process of reading, students prefer to summarize in their mother tongue, so as to establish a connection between the old information in their minds and the newly accepted information, and realize the integration of the old and new information [15].

The relationship between the amount of thinking in mother tongue and the difficulty of reading materials is shown in Table 4 after investigation and calculation. In CET-4 reading, mother-tongue thinking accounts for 59.0% of the total language thinking while the participation of mother-tongue thinking in CET-6 reading is 54.5%. The abovementioned data seem to indicate that students tend to use their mother-tongue thinking to help understand the text when reading low-difficulty texts. However, after careful observation, it can be seen that when the amount of independent thinking in English changes little (3.7% and 2.9%, respectively), the proportion of English used for reading text increases from 37.3% to 42.6%, and the proportion of English used for reading increases. It is also inevitable that the amount of mother-tongue thinking participation decreases.

### 4.4. Conclusion

On the whole, non-English majors are involved in mother-tongue thinking to a great extent in the process of English reading comprehension, and thus carry out various thinking activities [16]. In the process of reading, the mother tongue is often used not only to summarize the text content, translate English directly into the mother tongue, and evaluate the text content, but also to associate information outside the text and measure the degree of self-understanding. When college students read texts with different degrees of difficulty, the participation of mother-tongue thinking has little change in quantity, but there are obvious differences in function; in the process of reading texts with low degrees of difficulty, students tend to use their mother tongue to associate the content outside the text and evaluate the content of the text. When dealing with difficult texts, they often use more mother-tongue thinking to summarize the text, guess the meaning of words and sentences, and give self-feedback on whether the meaning of the text is understood or not. In terms of specific thinking activities, students rely more on mother-tongue thinking when commenting on the information contained in difficult texts and evaluating reading results, especially when summarizing low-difficulty texts.

## 5. The Distribution and Types of Chinese-English Nominalization in Political Discourse and Its Translation

This chapter mainly makes an overall survey of the distribution and types of Chinese-English nominalization in political discourse and its translation, and makes a multidimensional analysis of the distribution, syntactic, and semantic features of Chinese-English derived, transferred, and phrase nominalization structures. This chapter attempts to find the distinctive and regular features of the use of Chinese and English nominalization in political discourse and its translation from the perspective of use and quantitative analysis. Statistics on the Chinese source database and the English translation database show that nominalization has a high frequency of use in political discourse and its translation, which is a common lexical and grammatical feature of Chinese and English political discourse. Different types of nominalization have significant differences in the use of Chinese and English [17].

### 5.1. Chinese-English Nominalization and Its Translation Strategy Distribution

In order to more intuitively understand the use of nominalization in political discourse and its English translation, we annotated Chinese and English nominalization in a sample of 1000 nominalization sentence pairs according to the classification criteria and counted the distribution characteristics of various types of Chinese-English nominalization, as well as the distribution characteristics of their equivalence and transfer translation strategies.

Table 5 shows the distribution of Chinese and English nominalizations in the sample. The overall frequency statistics show that the frequency of nominalization in English target discourse is about 1.5 times that in Chinese source discourse, but in proportion, the two are close to the same [18]. This result shows that the target text basically maintains the same metaphorical degree as the source text, and that nominalization is not the exclusive product of English political discourse. The proportion of nominalization in Chinese political discourse is equivalent to that in English, which deserves academic attention and attention, especially the large number of nominalization phenomena used flexibly in the structure.

In addition, there are obvious differences in the distribution of different types of nominalizations between Chinese and English.  Figure 9 compares the proportions of various types of nominalizations in Chinese and English in the expression of nominalization in corresponding languages. The figure clearly shows the differences in the structure and use preferences between Chinese and English nominalization. As shown in Figure 9, there are great differences between the two languages in the use of derived and trans-type nominalization. The vast majority of Chinese nominalization is trans-type (87.4%), while English nominalization is mainly derived type (82.8%). The chi-squared test shows that the use of English-derived nominalization is significantly higher than that of Chinese-derived nominalization (*X*^2^-1303.2, *p*=000), while the use of Chinese turn-type nominalization and phrase-type nominalization is significantly higher than that of similar English nominalization (*X*^2^ = 1361.9, *X*^2^ = 72.7, *p*=.000). From the absolute value of the chi-squared test, the conversion type nominalization is the main source of the differences in the use of nominalization between the two languages, followed by the derived type, and the phrase type nominalization has the smallest difference [19].

Figure 10 shows the corresponding situation of Chinese-English nominalization in the sample corpus from the perspective of translation. It can be clearly seen from the pie chart that nearly half of the 3297 correspondences containing nominalization are nominalized equivalent translations, which shows that translators tend to retain the same way of understanding the original text in order to pursue stylistic equivalence in political text translation.

In addition, we also made statistics on the specific corresponding contents of nominalization in the two transfer translation directions (Figure 11). As can be seen from the figure, the nominalization structure mainly corresponds to other types of phrases at the same level, such as common noun phrases, verb phrases, and adjectives. The transformation between verb phrases and adjective phrases, and the nominalization structure is more in line with the expectation, which can be compared with the transformation relationship between congruence and metaphor. The transformation in the process of translation is inevitably related to the collocation habit of the language expression and the translator's subjective role.

### 5.2. Chinese-English-Derived Nominalization

There are great differences between Chinese and English in the types, productivity, nominalization, and semantic emptiness of the derived affixes, as well as the nominalized affixes. Since the formal markers of Chinese- and English-derived nominalization have the overall quantitative conditions, we have identified and quantified all derivatives in the corpus. The results show that there are 1210 Chinese derivatives in the corpus and 29859 English derivatives. From the frequency of use, the frequency of derived nominalization in English target discourse is about 24 times that in Chinese source discourse. According to Figure 12, the observed Chinese-derived affixes reflect the derivation ability of different affixes. In terms of derivational nominalization, the diversity, productivity, and stability of English nominalized derivational affixes are better than those of Chinese, and there are obvious differences in their composition and use. However, Chinese-derived affixes do not have the function of marking parts of speech like English affixes. The same derived word can also have the use of verbs or adjectives in addition to acting as a noun [20].

### 5.3. Text Complexity Feature Extraction

The “absolute complexity” of text is the focus of this study. It originates from the language units in the text and belongs to the complexity of the objective internal characteristics of the language system. For example, the number of specific components of a language feature or language system, the number of relationships between different components, and so on. In this study, we define the operationalization of text complexity features as “a text complexity index that can be automatically extracted by software or programs and does not vary from person to person,” and examine the text complexity from the following three dimensions: vocabulary, syntax, and discourse. The number of cohesion indicators in COH-metrix is relatively limited. It only involves local cohesion between sentences (such as content word overlap between sentences) and overall cohesion (such as the number of all pronouns and conjunctions in the text). It does not consider the overall cohesion of large text units (such as argument overlap between paragraphs). Moreover, there is a high degree of collinearity between the cohesion indicators provided by COH-metrix. In contrast, TAACO includes three types of indicators: local, overall, and full-text cohesion. Based on the abovementioned considerations, this study will use TAACO 2.0 as a tool to extract text complexity information from textbooks. Specifically, the cohesive features in TAACO can be divided into the following five categories: connectives, knowability, type ratio, lexical overlap, and semantic similarity.

The essence of principal component analysis is the rotation transformation of coordinates. The original *n* variables are relinearly combined to generate *n* new variables. They are not related to each other and are called *n* “components.” At the same time, the principle of “variance maximization” ensures that the variance of the first component is the largest, and then decreases in turn. These *n* components are arranged in the order of variance from large to small, and the first *m* components may contain most of the variance (and variation information) of the original variables. Then, these *m* components become the “principal components” of the original variables, and they contain most of the information of the original variables [21].

It can be calculated according to the transformation of x1- and x2-related variable vectors y1- and y2-unrelated variables.

(1) $$\begin{array}{c} Y1={\frac{\text{sqrt}2}{2}}^{*}X1+{\frac{\text{sqrt}2}{2}}^{*}X2,\\ Y2={\frac{\text{sqrt}2}{2}}^{*}X1+{\frac{\text{sqrt}2}{2}}^{*}X2, \end{array}$$

where sqrt (*x*) is the square root of X. Through the relinear combination of *X*1 and *X*2, two new variables *Y*1 and *Y*2 are obtained. At this time, *Y*1 and *Y*2 are no longer relevant, and the variation variance in the *Y*1 direction is large, but the variation variance in the *Y*2 direction is small. At this time, *Y*1 can be extracted as the principal component of *X*1 and *X*2 to participate in the subsequent statistical analysis, because it carries most of the information of the original variables. After this operation, the purpose of reducing the dimension and eliminating collinearity is achieved.

In the process of verification, a neural network can be used to calculate and identify the information with the simplest feedforward neural network (Figure 13): *Y*(*n*)=[*y*_1_(*n*), *y*_2_(*n*),…,*y*_1_(*n*)]^*T*^ is the input vector. $\bar{X}\left(\text{n}\right)={\left[{\tilde{X}}_{1}\left(\text{n}\right),{\tilde{X}}_{2}\left(\text{n}\right),\ldots ,{\tilde{X}}_{\text{k}}\left(\text{n}\right)\right]}^{T}$ is the output vector.

There are usually two methods for model evaluation: data-driven or user-based. Under the data-driven paradigm, prediction accuracy and other indicators are usually used to evaluate the model; under the user-based paradigm, the evaluation usually depends on the readers' recall and understanding of texts with different complexity. As mentioned before, the object of this study is absolute complexity independent of users, so the data-driven method is used to evaluate the model. The common performance metrics in classification model evaluation are precision (P), recall (R), accuracy (a), and F-measure (F-measure). The recall rate, accuracy rate, and F-measure value of the text classification model are calculated using the following formulae:

Accuracy: *p*=*Tp*/(*Tp*+*FP*)^*∗*^100%; the accuracy rate describes how many of the identified results in the classification model are classified into correct categories from the perspective of prediction.

Recall rate: r=*Tp*/(*TP*+*FN*)^*∗*^100%; recall rate describes how many texts have been correctly recognized by the classification model from the perspective of real results.

Accuracy: a=(*TP*+*TN*)/(*TP*+*FP*+*FN*+*TN*)^*∗*^100%; accuracy refers to the proportion of the number of texts correctly recognized by the classification model to the total number of recognized entities.

F-measure value: *Fβ*=(*β*^2^+1)^*∗*^p^*∗*^r/(*β*^2^ ^*∗*^p+r), where *β* is the parameter that adjusts the proportion of the correct rate and recall rate in the evaluation function. Usually, *β* = 1. The evaluation index at this time is simplified as follows: *F*1=2^*∗*^p^*∗*^r/(p+r).

Generally, the research will report the recall rate (*R*) and the accuracy rate (P), but sometimes they are contradictory, which requires comprehensive consideration. The most common method is the F-measure, also known as the F-score, which is the weighted harmonic average of the accuracy rate and the recall rate. When the parameter *b* = 1, it is the most common *F*1, which combines the accuracy rate and the recall rate. Generally, when multiple model assumptions are compared, the higher the *F*1 value is, the more effective the classification model is. Therefore, this study mainly reports the recall rate, accuracy rate, and *F*1 value of the model.

## 6. Conclusion

From the perspective of functional linguistics, under the framework of the reinstantiation model of the translation process, and based on the theory of grammatical metaphor, this paper makes a systematic study of political discourse and its Chinese-English nominalization in translation. Based on the self-built Chinese-English parallel corpus of political discourse, this paper makes a qualitative and quantitative analysis of the distribution and type characteristics of Chinese-English nominalization, translation equivalence, and transfer mode, summarizes the translator's methods and regular characteristics of dealing with the expression of Chinese-English nominalization, discusses the influencing factors and construction functions of the nominalization translation mode in political discourse from various dimensions, and reveals the significant potential of well-known nominalization in cross-language reinterpretation. This paper mainly summarizes the research findings, explains the main contributions and enlightenment of this study, and reflects on the limitations and the research space of this study.

The limitation of the scope of the study lies in the inability to take into account multiple genres, translation directions, and translations at the same time. The genre observed in this study is political discourse, which is not covered in other types of discourse. Nominalization and its translation should have different construction functions and translation rules in literary discourse, academic terminology discourse, scientific discourse, and legal discourse. In addition, the corpus observed in this study only includes one translation direction of Chinese-English translation, and lacks two-way parallel observation and comparison of English-Chinese texts. In addition, since most of the published English versions of political discourse are authoritative official versions and cannot be compared with multiple versions, the translator's subjectivity has not been fully explained. By comparison with student translators or senior translators, the investigation and interview with translators or target language readers are increased, and the translation research of political discourse and the application value of the research can be enriched. The follow-up studies should give further play to the theoretical advantages of functional linguistics as applicable linguistics and create more space for the study of the translation theory and translation description.

## Figures and Tables

**Figure 1:** Culture, meaning, and scenario.

**Figure 2:** Schematic diagram of the relationship between genre and style.

**Figure 3:** Definition of business English.

**Figure 4:** Hierarchy of international business languages.

**Figure 5:** Grammatical metaphor as tension between language levels.

**Figure 6:** Formation diagram of the language knowledge structure and cognitive structure.

**Figure 7:** Relationship between the mother-tongue knowledge structure and cognitive structure.

**Figure 8:** Relationship between knowledge structure and cognitive structure of mother tongue and English.

**Figure 9:** Comparison of Chinese and English nominalization types.

**Figure 10:** Distribution of nominalization equivalence and transfer translation strategies.

**Figure 11:** Translation types of nominalization transfer.

**Figure 12:** Productivity statistics of Chinese-derived affixes.

**Figure 13:** Structure diagram of the feedforward neural network.

**Table 1:** Description of reading text features.

	Total words	Average word length	Total sentences	Average sentence length
CET-4	229	4.7	9	25.4
CET-6	400	5.4	21	19.2

**Table 2:** Mother tongue and English thinking participation in reading.

Total words	Number of Chinese words (%)	Number of English words (%)	
		Repeat reading material statements	Autonomous thinking
1318	740 (56.2%)	535 (40.6%)	45 (3.2%)

**Table 3:** Mother tongue and English thinking participation in reading.

Classification of mother-tongue thinking activities			Mother-tongue thinking amount (%)
Meaning level thinking activities635 (85.2%)	Literal comprehension 163 (21.8%)	Literal translation	140 (18.8%)
		Semantic guessing	23 (3.0%)
	Inferential understanding 379 (50.8%)	Forecast below	22 (2.8%)
		Extension of literary meaning	43 (5.7%)
		Summary of text and meaning	203 (27.6%)
		Literary and semantic association	110 (14.7%)
	Evaluative comprehension		93 (12.6%)

Formal thinking 58 (7.2%)	Word analysis		9 (0.9%)
	Sentence analysis		27 (3.4%)
	Paragraph analysis		22 (2.9%)

Self-management level thinking activities 59 (7.6%)	Process monitoring		1 (0.7%)
	Process adjustment		22 (2.8%)
	Understanding assessment		31 (4.1%)

Total			752 (100%)

**Table 4:** Mother tongue and English thinking participation in reading high-and low-difficulty materials.

Reading materials	Total words	Number of Chinese words (%)	Number of English words (%)	
			Repeat reading material statements	Autonomous thinking
CET-4	1010	596 (59.0%)	374 (37.3%)	40 (3.7%)
CET-6	1621	884 (54.5%)	690 (42.6%)	47 (2.9%)

**Table 5:** Basic information on the frequency of nominalization in Chinese original text and English translation.

Language	Sample size (shape symbol)	Nominalization type and frequency				
		Derived type	Transfer type	Phrasal type	Population	Proportion (%)
Chinese nominalization	20.162	169	1732	80	1981	9.84
English nominalization	29.346	2391	476	20	2887	9.83
	*X * ^2^	−1303.2	1361.9	72.7		
	*p*	000	000	000		

## Data Availability

The labeled data set used to support the findings of this study is available from the author upon request.
